# Analysis of Characteristic Factors of Nursing Safety Incidents in ENT Surgery by Deep Learning-Based Medical Data Association Rules Method

**DOI:** 10.1155/2022/8491411

**Published:** 2022-10-12

**Authors:** Ju Chen, Jie Zhou, Fanglan Yang

**Affiliations:** Anesthesia Operation Center, 363 Hospital, Chengdu, Sichuan 610041, China

## Abstract

It is of great significance to explore the characteristic factors of postoperative nursing safety events in patients with otolaryngology surgery and to understand the characteristics of postoperative nursing safety events in otolaryngology surgery patients. This paper carried out preoperative safety protection for 385 inpatients, and the results showed that there were 52 cases of postoperative safety nursing events. This experiment found that the coinfected lesions (*P* = 0.001, HR = 14.283, 95.0% C1: 9.365~21.038), the treatment period (*P* = 0.001, HR = 13.716, 95.0% CI: 7.147~20.275), during hospital treatment (*P* = 0.002, HR = 15.208, 95.0% CI: 8.918-24.237), antibiotic use (*P* = 0.001, HR = 14.054, 95.0% CI: 8.163-21.739), and hypertension (*P* = 0.001, HR = 13.976, 95.0% CI: 7.926-22.385) are the important factors affecting postoperative care; using the association rule method to control and analyze the main risk factors of postoperative infection and bleeding in ENT patients can significantly improve the prognosis.

## 1. Introduction

Since the discussion of data mining and knowledge discovery first appeared in the world, the current data mining technology has been quite perfect [1]. Data analysis technology is the continuous improvement of data processing and analysis capabilities, which can quickly discover valuable knowledge. Data mining technology and software have been widely used in all walks of life and have produced significant economic and social benefits in medical and health care. However, the application in healthcare is still in its initial stage. Compared with other industries, the healthcare industry needs data mining technology for data processing, and this industry can perform auxiliary examinations, experience summaries and data analysis after using this technology. Therefore, medical data mining has more practical significance. Development prospects [2] in medical research, the extensive application of data mining technology in medicine will be recognized by more medical institutions and personnel. The particularity, timeliness, complexity, instability, and incompleteness of medical data. At present, the urgent problem to be solved in the processing of medical data is how to mine useful information from the data. These research results can play an important role in the diagnosis and treatment of diseases, the scientific decision-making of medical and health management departments, the epidemic of diseases, the prevention and treatment of infectious diseases, and health examinations [3–5]. Through research on the application of clinical and medical drugs, common clinical methods can be found to rationally use drugs for clinicians and reduce the physical and psychological burden of patients. If the means and means of data processing can be used to discover hidden, in-depth and diagnostically valuable data and rules from the massive data, and transform these massive data into valuable wisdom, it will greatly improve the hospital and the ability of medical workers to diagnose and treat, reduce the rate of misdiagnosis, and reduce the physical, mental, and financial pressure of patients. Due to the increasing popularity of computer science and technology, the amount of data required by various disciplines has increased dramatically. Therefore, how to find useful information from a large amount of data needs to be analyzed through data mining technology. During the development of association law, this new method was used to conduct in-depth discussions on clinical disease monitoring, drug treatment effect evaluation, and disease prevention and treatment.

The safety of nursing is generally the absence of any mental, structural or functional impairment, handicap, defect, or lethality throughout the duration of medical care [6]. The work of nurses is complex, involves a wide range of areas, and has many reasons for instability, which will not only have a great negative impact on the quality of nurses' work but also have a negative impact on the hospital's society and economy. In recent years, nursing workers have been accumulating and accumulating experience in their work to improve the level of nursing safety, prevent the occurrence of medical safety incidents, enable patients to receive appropriate, timely and safe nursing care, and maintain and restore the patient's body.

Otolaryngology is a relatively common disease, and complications such as infection and massive bleeding often occur during surgery, which pose a great threat to the survival of patients [7]. There are several main reasons that affect the safety of nursing care of surgical patients [8]. This therapy not only brings more pain to the patient but also brings greater financial pressure to the patient. Taking appropriate nursing measures can prevent and reduce postoperative complications as soon as possible [9].

In this paper, 385 otorhinolaryngology surgical patients from October 2019 to December 2021 were selected as the survey subjects, using the deep learning-based medical data correlation rule method and using the single factor analysis and logistic variance regression methods to carry out the statistics of risk factors. The purpose is to provide a certain reference for the nursing safety of patients undergoing ENT surgery in clinical practice.

## 2. Introduction to Related Theories

### 2.1. Data Mining Based on Deep Learning

Data mining (DM), also known as KDD, is a new information processing technology emerging in recent years [10]. DM is to extract implicit, regular, unknown, but potential and understandable information or models from massive data in databases, data warehouses, or other databases [11]. DM is based on database technology, which organically integrates artificial intelligence, parallel computing, statistics, and neural networks. Data mining is a process that uses a variety of analytical methods to discover patterns and connections between data from a large amount of data, and use this to make predictions and help decision makers find possible connections between data and find possible overlooked connections. Therefore, it has become an effective means to deal with the current explosion of data and the lack of information.

DM can discover potential, novel, effective, easy-to-understand, and easy-to-store, and apply knowledge techniques and approaches from massive data [12]. DM does not need to establish accurate retrieval requirements when dealing with massive data and converts massive data into meaningful information to describe the trend of historical development, respond to future development directions, obtain effective query performance, and provide support for decision-making news. Data mining is to unearth some hidden, unknown in advance but potential, and unearthed into rules, patterns, and other forms from the data warehouse.

The modes of data collection are as follows: classification model, regression model, and time series model are all model-based. The model consists of clustering model, association model, and sequential model.

The method first describes a predetermined set of data or concepts, and then models the database unit, assuming that the unit is a predetermined category, the unit is called a “class”; the units are called “class sets” and are “sampled” for said “training” selection;

The continuity of the regression model was simulated using multiple regression statistics. Many problems can be solved by linear regression, and nonlinear problems can be transformed into linearization to solve.

The time series model is to use the time series trend of the existing data to predict it. This is very similar to the linear regression model. However, timing analysis must take into account the time domain characteristics, especially the impact on the time domain. On this basis, in order to accurately predict the future values, the influence of time must be fully considered, and a dynamic analysis of a set of values must be carried out according to the existing data.

The cluster mode is to divide a population into several categories, so that the populations of the same population are as close as possible, while the number of populations between various groups is minimized. Combining a group of entities or a group of abstract objects into multiple categories of similar objects is called cluster mode, which is decomposed and merged according to specific cluster parameters. Once the purpose is achieved, the category parameters can be obtained by this method.

### 2.2. Association Rules

The data mining method of association law is divided into two stages: looking for the shortest number of occurrences (testing of the degree of support); based on the strong correlation criterion (CI) generated by the collection of current items, it needs to meet the least degree of support and the least credibility.

The first step is the most important, and its effectiveness is directly related to the overall effect of data mining. For better understanding, the algorithm for data collection should be as simple as possible. In order to test the correctness of the relevant criteria, this paper uses the support degree and credibility of the association criterion to measure its weight, and its promotion degree to measure its importance. Indicators such as support, confidence, and improvement of association criteria cannot only measure the quality of relevant criteria but also a key factor to measure the formulation of association criteria.

### 2.3. Association Rules Apriori Mining Algorithm

On this basis, Hongli et al. implemented a new data mining method using the Apriori algorithm [13]. The method can reduce the storage capacity of the database, increase the utilization rate of the system, and can find frequent items and discover the deeper rules.

If the item set l is a regular item set, then all its nonempty item sets must also be a regular item set. If a (*k* + 1)-item set is a frequent item set, then all its k-item sets must also be a frequent item set. On the contrary, if the k-item set is not a frequent item set, then all the k-item sets in the item set must be frequent itemsets. The (*k* + 1)-item set is not a frequent itemset, so during the step-by-step retrieval, the generation of the frequency (*k*+ 1)-item can be realized by methods such as connection, pruning, and auxiliary statistics.

## 3. Application Method Design

### 3.1. Research Objects

From October 2019 to December 2021, a total of 385 otolaryngology patients aged 17-73 in a hospital were selected, with an average of (47.8 + 13.2). Of these patients, 190 were men, and 195 were women. All patients underwent ENT surgery and were excluded. 264 patients also had hypertension. Postoperative care was given to 52 patients who had undergone otolaryngology surgery.

### 3.2. Methods

Risk factors such as gender, age, infection site, pathogen type, operation time, hospital stay, antibiotic use, and hypertension were collected in this experiment. All cases were followed for one year to determine the presence of comorbidities and recurrence.

### 3.3. Association Rules Method

Weka mining software was selected for this study. Weka, fully named Waikato Intelligent Analysis Environment, is a java-based open-source product for data mining and knowledge discovery.

Weka is one of the most complete data mining tools available today and is recognized as the most famous open source product for data mining. It provides a unified user interface and integrates a large number of machine learning algorithms that can undertake data mining tasks, including preprocessing of data, association rule mining, classification, clustering, etc., and provides rich visualization capabilities. At the same time, due to the openness of its source code, Weka cannot only be used to complete the regular data mining tasks but also can be used for secondary development of data mining. As shown in Figure 1.

Data processing and transformation: web mining data comes in the form of arff files. First, save the marriage inspection data in the form of an Excel file, save the worksheet into a.csv file, then go to the Weka exploration program Explore, open the csv file, and then save it as an arff file, as shown in Figure 1 for the transformation of the file. Input the data into the data mining software Weka, convert it into the Associate label, click the “Choose” button, select Apriori, set minsupport = 30%, minconfidence = 80%, establish the relevant relationship, and click the “Start” button to start mining.

### 3.4. Statistical Processing

Used to conduct statistics on all data, and the measured values were expressed as (&- + s). The count data were tested by using *t*-test for comparison, and multifactor logistic regression was carried out for the variables with important influence, *P* < 0.05 shows a significant difference.

## 4. Analysis of Applied Practice Experiments

### 4.1. Univariate Regression Analysis

Statistics show that operative time, intraoperative bleeding and length of hospital stay are the main factors affecting postoperative complications. In the statistical data, the use of antibiotics, the combination of hypertension, the site of infection, and whether there is blood transfusion during the operation are the main reasons that affect the complications of surgery. The above risk factors were significantly different among the risk factors in ear, nose, and throat surgery (*P* < 0.05).(see Tables 1 and 2).

### 4.2. Multivariate Logistic Regression Analysis of Risk Factors

Risk factors for each factor were analyzed, and it was found that the intraoperative OR was 2.537, *P* = 0.023; the hospitalization time was 5.208, *P* = 0.003; the antibiotic use OR was 2.234, *P* = 0.028, and the intraoperative bleeding OR = 1.005, *P* = 0.001. Complicated with hypertension (OR = 2.013, *P* = 0.015), infection at the combined place (OR = 2.711, *P* = 0.013). See Table 3.

## 5. Conclusion

The three major types of ENT diseases include chronic otitis media, chronic tonsillitis, chronic sinusitis, nasal polyps, deviated nasal septum, acute and chronic laryngeal obstruction, ear, nasal cavity, sinus, and throat and neck tumors. Some ENT diseases require surgery, and nursing safety issues such as bleeding, infection, etc. are very common and can have a great negative impact on patient survival and survival. Lihua et al. [14] conducted a survey on 164 patients who had received ENT surgery, and the results showed that, on this basis, 14.02% of the patients had nursing safety problems. A total of 59 of 385 patients in this paper, of which 59 patients had nursing safety accidents after surgery, the incidence rate was 15.3%, which was in line with the above reported situation.

Nursing safety accidents that occurred after surgery not only aggravated the patient's condition but also caused the patient and their families to bear unnecessary economic pressure. Therefore, the analysis of the safety risk of postoperative nursing of stroke patients has an important guiding role in the treatment and prognosis of the disease. Multivariate logistic regression was used to analyze the effect of nursing safety after otolaryngology surgery, and the public analysis of 5 j was preliminarily discussed.

### 5.1. Operation Time

The duration of the operation is one of the main causes of postoperative infection, and as the operation progresses, the exposure time of the wound increases as the operation time goes on, and at the same time, as the operation continues, the postoperative bleeds. The amount and duration of anesthesia will also be greatly reduced, resulting in reduced patient tolerance, thereby increasing the infection rate of the wound surface, thereby greatly improving the safety of nurses. The survey results of Aghamohammadi et al. [15] showed that in ENT surgery, the incidence of nurse safety accidents within 30 minutes before the operation was 6%, and among patients with more than 30 minutes, 17.1% of the patients appeared nursing. On this basis, the postoperative treatment period (35.46 + 2.31) minutes of postoperative combined and noncombined patients had a significant effect on the treatment effect of 28.73 + 2.25 minutes (*P* < 0.05); the multiple linear regression results showed that the OR was 2.537, *P* = 0.023. Therefore, in ear, nose, and throat surgery patients, the duration of surgery is an important reason for the safety of nurses.

### 5.2. Length of Hospital Stay

With the development of hospitals, patients have more and more contact with hospital patients, more and more pathogenic bacteria on their bodies, and more and more close contact with patients and medical staff, making them more susceptible to pathogens, and these viruses are emitted from the air [16] . In this test, the days of admission for the combined and noncombined (5.69 + 0.61) were significantly compared with 4.67 + 0.56 d (*P* < 0.05); the multiple linear regression results showed that the difference between the two was significant OR was 5.208, *P* = 0.003. In conclusion, the length of hospital stay has a certain influence on the safety of nurses after surgery. However, if early intervention can reduce the recurrence after surgery, it remains to be further explored, and this trial is a single-point trial, involving a small number of patients, and has some limitations.

### 5.3. Intraoperative Blood Loss

Massive bleeding during surgery is unavoidable, but because blood will inhibit the body's immune system to a certain extent, this effect will cause strong resistance to cytokines, significantly increase the number and function of T lymphocytes, and also the response and response of lymphocytes to soluble antigens and mitogens, thereby inhibiting the normal killing of cells and increasing the safety of postoperative care. The results of multivariate regression showed that intraoperative blood loss was significantly associated with postoperative complications (OR = 1.005, *P* = 0.001). However, if you pay attention to enhancing the patient's immunity during blood transfusion, because intraoperative bleeding cannot be an important reason for affecting the safety of postoperative care in otolaryngology surgery, it is necessary to strengthen immunity during otolaryngology surgery to achieve purpose of prevention. At the same time, it is necessary to strengthen the technique of the surgeon, shorten the operation process as much as possible, reduce the postoperative blood loss rate, and ensure the standardization of the operation [17].

### 5.4. Antibiotic Use and Comorbid Hypertension

The application of various antibiotics will cause damage to the patient's body, which means that the living environment of microorganisms has been greatly affected, and at the same time, the bacteria will develop resistance, thus greatly increasing the infection rate of bacteria [17] . Hypertension is a relatively common complication in chronic rhinitis patients, especially in the elderly, and with age, the patient's physical functions are also affected. After logistic regression analysis, it was found that the OR of antibiotics was 2.234, *P* = 0.028, and the combined hypertension OR was 2.013, *P* = 0.015; the difference between the two was significant, suggesting that the use of antibiotics and hypertension during surgery is the main cause of nurses' safety incidents.

### 5.5. Infection Complicated Site

Patients in ear, nose, and throat surgery are mainly due to respiratory infections. These bacteria will invade the human body from the mouth and nasal passages. When the human body is weak, it is easy to cause some respiratory system problems, and some viruses will suddenly enter the digestive tract. Therefore, in this trial, the probability of safety events in patients with postoperative respiratory care was 24%, which was significantly different from other wards.

The independent risk factors of postoperative nursing safety of ENT patients can guide doctors to control the risk factors of various nursing safety events during surgery. Clinical data of patients in the department of ENT, using deep learning-based medical data association rules method, univariate analysis and logistic regression to analyze the risk factors of postoperative nursing safety events in patients with ENT surgery, and the research results on postoperative infection and bleeding in ENT patients. The main risk factors can significantly improve the prognosis. Effectively reduce the occurrence of nursing safety incidents and improve patient prognosis. Of course, there are some problems in the research process. The sample size of this study is still small, and the collection and comparison of clinical data is not comprehensive.

## Figures and Tables

**Figure 1:** Weka software interface.

**Table 1:** Statistical *t*-test analysis of postoperative safety nursing factors for ENT patients.

Risk factors	(Age)	Operation time (time)	Length of hospital stay (d)	Intraoperative blood loss (mL)
Uncomplicated group (*n* = 326)	57.36 ± 5.67	28.73 ± 2.25	4.67 ± 0.56	46.52 ± 13.17
Complication group (*n* = 59)	58.77 ± 5.61	35.46 ± 2.31	5.69 ± 0.61	756.23 ± 20.65
*t* value	1.7605	21.0556	12.6960	53.4361
*P* value	0.0791	0.001	0.001	0.001

**Table 2:** Test and analysis of count data of nursing safety factors after ENT surgery *x*^2^.

Risk factors		Number of cases	Complications (cases)	*x* ^2^ value	*P* value
Infection concurrent site	Respiratory tract	179	43	18.184	0.001
	Urinary system	69	5		
	Digestive tract	83	6		
	Other	51	6		
Gender	Male	191	29	0.004	0.948
	Female	194	30		
Types of germs	Gram positive	203	31	0.012	0.912
	Gram negative	182	28		
Intraoperative blood transfusion	Have	73	48	171.775	0.001
	None	312	11		
Antibiotic use	Have	337	56	4.067	0.044
	None	52	3		
Hypertension	Have	271	53	11.557	0.001
	None	114	6		

**Table 3:** Multivariate logistic regression analysis of nursing safety factors after ENT surgery.

Risk factors	Partial regression coefficient	Standard deviation	OR	*P* value	Wald	95% confidence interval
Infection concurrent site	0.995	0.402	2.711	0.013	6.1174	1.229~5.867
Operation time	0.936	0.425	2.537	0.023	.736	1.103~5.931
Hospital stay	0.985	0.763	5.208	0.003	5.208	1.172~3.830
Intraoperative blood loss	0.004	0.001	1.005	0.001	16.608	1.002~1.006
Antibiotic use	0.833	0.372	2.234	0.028	4.271	1.079~3.267
Hypertension	0.702	0.284	2.013	0.015	6.017	1.149~3.521
Constant	0.506	1.136	1.662	0.661	0.192	

## Data Availability

The dataset used in this paper are available from the corresponding author upon request.
